# Big Data Analysis and Application of Liver Cancer Gene Sequence Based on Second-Generation Sequencing Technology

**DOI:** 10.1155/2022/4004130

**Published:** 2022-08-16

**Authors:** Chaohui Xiao, Fuchuan Wang, Tianye Jia, Liru Pan, Zhaohai Wang

**Affiliations:** ^1^Faculty of Hepato-Biliary-Pancreatic Surgery, Chinese People's Liberation Army (PLA) General Hospital, Beijing 100853, China; ^2^Faculty of Hepatology Medicine, Chinese People's Liberation Army (PLA) General Hospital, Beijing 100039, China; ^3^Department of Laboratory, Fifth Medical Center, Chinese People's Liberation Army (PLA) General Hospital, Beijing 100039, China

## Abstract

In big data analysis with the rapid improvement of computer storage capacity and the rapid development of complex algorithms, the exponential growth of massive data has also made science and technology progress with each passing day. Based on omics data such as mRNA data, microRNA data, or DNA methylation data, this study uses traditional clustering methods such as kmeans, K-nearest neighbors, hierarchical clustering, affinity propagation, and nonnegative matrix decomposition to classify samples into categories, obtained: (1) The assumption that the attributes are independent of each other reduces the classification effect of the algorithm to a certain extent. According to the idea of multilevel grid, there is a one-to-one mapping from high-dimensional space to one-dimensional. The complexity is greatly simplified by encoding the one-dimensional grid of the hierarchical grid. The logic of the algorithm is relatively simple, and it also has a very stable classification efficiency. (2) Convert the two-dimensional representation of the data into the one-dimensional representation of the binary, realize the dimensionality reduction processing of the data, and improve the organization and storage efficiency of the data. The grid coding expresses the spatial position of the data, maintains the original organization method of the data, and does not make the abstract expression of the data object. (3) The data processing of nondiscrete and missing values provides a new opportunity for the identification of protein targets of small molecule therapy and obtains a better classification effect. (4) The comparison of the three models shows that Naive Bayes is the optimal model. Each iteration is composed of alternately expected steps and maximal steps and then identified and quantified by MS.

## 1. Introduction

Next-generation sequencing (NGS), also known as high-throughput sequencing or massively parallel sequencing, is a technology that can sequence thousands to billions of DNA fragments simultaneously and independently. The dideoxynucleoside end-termination sequencing method began in the 1970s. In the follow-up continuous improvement, the Sanger method caused a sequencing boom and became the mainstream due to its simplicity and rapidity. In order to meet the increasingly complex research needs, next-generation sequencing technology emerges from time to time [1–3]. Using NGS technology to detect a variety of cancers, and compared the results with the Sanger method, it was found that in addition to common gene mutations, NGS technology can also detect many gene mutations that were ignored by real-time quantitative PCR detection technology. It may play a prompting and guiding role in the occurrence and development of cancer and the diagnosis and treatment of patients and also reflects the value of using NGS technology in clinical work. There are currently three mainstream NGS platforms: Roche454, Ion Torrent, and Illumina platforms. The Roche454 platform is based on the pyrosequencing method, that is, bases are incorporated in the order of T, A, C, and G during sequencing, and pyrophosphate is released after pairing. The Ion Torrent platform is the semiconductor sequencing technology. The ion sensor can detect the pH change caused by proton release during the synthesis process and then judge the sequence of the base. NGS technology detection programs have different focuses, including whole genome sequencing (WGS), which can detect all genetic changes and conduct a comprehensive analysis of tumor-related genes, but it is costly and time-consuming. Whole exome sequencing (WES), which only detects the coding gene regions, is more economical and can detect already known mutant coding genes and discover new gene mutations in cancer. Whole transcriptome sequencing, based on cDNA sequence sequencing, can detect information about the overall transcriptional activity [4]. Targeted target sequencing can select some genes required for disease research for higher sequencing efficiency, but it is not suitable for detecting unknown mutations [5–7]. The techniques of experimental manipulation (wet experiment) and bioinformatics analysis (dry experiment) have been developed continuously. NGS technology is widely used in solid tumors, and more new gene mutations have been discovered, providing new ideas for the detection of genetic susceptibility and the guidance of individualized precision medicine, and have played an extremely important role in the study of the genetic pathways of human malignant tumor mutations effect. Liver cancer is one of the most common cancers in cancer patients today [8–10]. According to the 2020 report by the American Cancer Society, there are an estimated 42,810 new cases and 30,160 deaths from the liver and intrahepatic cholangiocarcinoma in the United States throughout the year. Statistics at home and abroad show that liver cancer is an important cause of cancer death worldwide, and the treatment of liver cancer is also an urgent problem to be solved. Liver cancer is divided into two types: primary and secondary. Primary liver cancer (PLC) is the most common. From a histological point of view, primary liver cancer can be divided into different subtypes according to the cell origin, hepatocellular carcinoma (HCC) (about 75-85% of all cases), intrahepatic cholangiocarcinoma (ICC) (about 75% of all cases), intrahepatic cholangiocarcinoma (ICC) (10-15%), and other rare forms. Hepatocellular carcinoma has become the main type of liver cancer research. The main known carcinogens of liver cancer are hepatotropic virus: mainly chronic infection with hepatitis B (HBV) and hepatitis C (HCV) virus; chemical stimulation: such as alcohol abuse and aflatoxin; metabolic abnormalities: diabetes and nonalcoholic fatty liver disease, hereditary hemochromatosis, etc.; immune-related causes: such as cirrhosis-related immune dysfunction syndrome (CAID) and autoimmune hepatitis; etc. Among them, viral infection is the main factor causing liver cancer [11–13]. Hepatocellular carcinoma cells have extensive heterogeneity from undesired lesions caused by a small number of mutations to eventually develop into an advanced form of the disease. Because the factors that induce liver cancer are diverse and the distribution in different countries and regions is different, the molecular mechanism of liver cancer is complicated. In a broad sense, liver cancer is divided into two categories: proliferative and nonproliferative. The proliferative type is common in HBV-induced liver cancer, with low degree of differentiation, high alpha-fetoprotein (AFP) expression, more vascular invasion, and worse prognosis; this type of liver cancer is characterized by increased inactivating mutations in TP53 and AXIN1, and at the same time, cell cycle, mTOR, RAS-MAPK, and MET signaling pathways that promote survival are all activated. The nonproliferative class is commonly seen in HCV and alcohol-related hepatocellular carcinoma, with moderate or high differentiation, low AFP expression, less aggressiveness, and chromosomal stability. This type of hepatocellular carcinoma is characterized by more heterogeneity, higher frequency of CTNNB1 (*β*-catenin) activating mutations, and TERT promoter mutations, as well as activation of WNT and IL6/JAK-STAT signaling pathways. However, these commonly mutated genes TP53, AXIN1, CTNNB1, and TERT in liver cancer proved to be difficult to target [14, 15]. At present, liver resection and liver transplantation have become the main treatment methods for patients with early-stage liver cancer, and patients with intermediate-stage liver cancer are often treated with hepatic arterial chemoembolization and radioembolization, which can greatly prolong the survival of patients. However, due to the lack of specific symptoms and tumor biomarkers, most HCC patients are diagnosed at an advanced stage, so these curative treatments are not suitable. Sorafenib, a multi-receptor tyrosine kinase inhibitor, was identified as a therapeutic drug with survival benefits for patients with advanced liver cancer. Multiple drugs have since been shown to have clinical efficacy, including other RTK inhibitors such as lenvatinib, regorafenib, and cabozantinib. The liver is an important organ that removes toxins and regulates blood sugar, fat, and amino acid uptake. Similar to all cancers, the gradual accumulation of genetic and epigenetic changes in the liver, accompanied by a large number of metabolic changes, leads to abnormal proliferation of mature hepatocytes and the evolution of liver cancer.. Due to the high heterogeneity of liver cancer cells and the complex pathogenic factors caused by the involvement of various signaling pathways, it is clinically found that using a unified treatment regimen to treat all patients may have different curative effects and may even exacerbate symptoms. Therefore, “personalized medicine” is the development direction of contemporary treatment of liver cancer, and different therapeutic methods based on molecular and cell therapy have also been developed. The emerging molecular-level therapeutic strategies include molecular targeted therapy, targeted radionuclide therapy, and epigenetic modification-based therapy, which provide new strategies for the treatment of liver cancer.

## 2. Big Data Analysis of Liver Cancer

### 2.1. Disease Diagnosis of Omics Big Data

Cancer subtype classification methods based on omics data mainly include subtype classification methods based on single omics data and subtype classification methods based on multiomics data fusion. The former is based on an omics data such as mRNA data, microRNA data, or DNA methylation data and uses traditional clustering methods such as kmeans, K-nearest neighbors, hierarchical clustering, affinity propagation, and nonnegative matrix decomposition to classify samples. The results of subtype classification of cancer are obtained, as shown in Figure 1. With the development of related technologies, the collection of omics data has shown an explosive trend, and its acquisition cost has been greatly reduced. A large number of genomics, transcriptomics, proteomics, and other data of different cancer patients are given in the database headed by TCGA omics data. Since different omics data can describe the complex life process in cancer cells and the interactions between various molecules from different perspectives, the information is complementary, and the integrated analysis of multiomics data can identify more accurate and reasonable subtype results. In recent years, research has mainly focused on the field of multiomics data integration analysis methods. Most existing integrative analysis methods need to address problems closely related to biological data. The data sample size is small, and the dimensionality is high (the so-called curse of dimensionality problem). When the data scope and data type are not consistent, the underlying omics-specific and between-group data structures are easily overlooked in multi-omics data. Divided from the data supported by integrative analysis methods, existing integrative analysis methods include general methods that can analyze any multiomics data and specialized methods designed only for specific data types. The former can be applied to any multiomics data and can be easily extended to the analysis of more omics data, while the latter requires the use of known biological relationships (such as the association between copy number changes and gene expression profiles), which can only be analyzed specific data types.

### 2.2. Epigenetics of Liver Cancer

Abnormal epigenetic changes are important etiologies for the occurrence, development, and metastasis of liver cancer. Epigenetics, the heritable modification of gene function without altering the DNA sequence, is caused by many different factors. Epigenetic alterations are often present in liver cancer. The screening process is shown in Figure 2. Epigenetic processes include, but are not limited to, chromatin remodeling, histone modification, DNA methylation, and expression of noncoding RNAs. Unlike the irreversible nature of genomic alterations, epigenetic changes are reversible, opening a promising avenue for the development of new therapeutic modalities. Therefore, epigenetic changes associated with cancer and liver cancer are gradually being widely used in the development of biomarkers. Hepatocellular carcinoma (HCC) is one of the most common liver tumors and has become the leading cause of cancer-related death in many regions and countries. Although many measures have been taken to prevent, early screen, diagnose, and treat liver cancer, the current situation of liver cancer in my country is still not optimistic.

## 3. Algorithm Model

### 3.1. Naive Bayes [16–20]

Semiconductor sequencing

(1) $$\begin{array}{c} X^{\prime }=\left\{\left(x_{1}^{\prime },y_{1}^{\prime }\right),\left(x_{2}^{\prime },y_{2}^{\prime }\right),\cdots ,\left(x_{n}^{\prime },y_{n}^{\prime }\right)\right\}X^{\prime }=\left\{\left(x_{1}^{\prime },y_{1}^{\prime }\right),\left(x_{2}^{\prime },y_{2}^{\prime }\right),\cdots ,\left(x_{n}^{\prime },y_{n}^{\prime }\right)\right\},\\ x_{\text{new}}=x_{i}+\mathrm{rand}\left(0,1\right)\times \left(x_{j}^{\prime }-x_{i}\right). \end{array}$$

Ion sensor, *D* is the matrix reconstruction function, *x* is the group sparse constraint function, and *y* is the weight of the group sparse constraint term.

(2) $$\begin{array}{c} D=\left\{\left(x_{1},y_{1}\right),\left(x_{2},y_{2}\right),\cdots ,\left(x_{m},y_{m}\right)\right\},\\ h_{i}=\varepsilon \left(N,m\right). \end{array}$$

Unknown genome sequence

(3) $$\begin{array}{c} H\left(x\right)=\arg_{\max}^{y\in Y}\overset{T}{\underset{t=1}{\sum }}\left(I\left(h\left(x\right)=y\right)\right.,\\ P_{i}=\left(x_{i},y_{i},z_{i}\right)\;i=1,2,3,4\cdots . \end{array}$$

Nucleic acid fragments are sequenced, *Row* is the number of clusters, *y*_*i*_ is the index of the sample belonging to the *i*th category, and *r* is the sparse constraint function.

(4) $$\begin{array}{c} \text{Row}=\frac{2y_{i}}{r},\\ \text{Column}=\frac{2x_{i}}{r}\;i=1,2,3,4\cdots ,\\ Z=\overset{n}{\underset{i=1}{\sum }}z_{i}. \end{array}$$

### 3.2. Okumura-Hata [21–23]

Assembly and splicing

(5) $$\begin{array}{c} X=\frac{\sum_{i=1}^{n}x_{i}z_{i}}{\sum_{i=1}^{n}z_{i}}. \end{array}$$

Coding gene regions for detection

(6) $$\begin{array}{c} Y=\frac{\sum_{i=1}^{n}y_{i}z_{i}}{\sum_{i=1}^{n}z_{i}},\\ L\left(db\right)=69.55-13.82\log h_{b}+\left(44.9-6.55h_{b}\right)\times \log d+26.16\log f_{c}-\alpha \left(h_{m}\right),\\ \alpha \left(h_{m}\right)=\left(1.11\log f_{c}-0.7\right)h_{m}-\left(1.56f_{b}-0.8\right),\\ \gamma \left(f_{c}\right)=8.29{\left(\log1.54h_{m}\right)}^{2}-1.1. \end{array}$$

Capture probe hybridization

(7) $$\begin{array}{c} f=3.2{\left(\log11.75h_{m}\right)}^{2}-4.97. \end{array}$$

Quality control

(8) $$\begin{array}{c} C_{\text{cell}}=-2{\left[\log\left(\frac{f_{c}}{28}\right)\right]}^{2}-5.4. \end{array}$$

Data filtering

(9) $$\begin{array}{c} \sigma_{\text{cell}}=-4.78{\left(\log f_{c}\right)}^{2}-18.33\log f_{c}-40.98,\\ P\left(dB\right)=13.82\log h_{b}+\left(44.9-6.55\log h_{b}\right)\times \log d+33.9\log f_{c}-\alpha \left(h_{m}\right). \end{array}$$

### 3.3. AdaBoost [24–27]

(10) $$\begin{array}{c} L\left(dB\right)=k_{1}+k_{2}\log d+k_{3}\log h_{b}+k_{4}{Diff}_{\text{loss}},\\ x_{i}=\max\left(B\_loc_{i},B\_Bore_{i}\right). \end{array}$$

For sequence alignment, *f*_*i*_ is a shared implicit expression matrix, and *x*, *k* are modality-specific basis matrices.

(11) $$\begin{array}{c} f_{i}=\text{SPM}\left(x_{i},k_{1},k_{2}\right),\\ \langle k_{1},k_{2}\rangle =\text{argmin}\overset{N}{\underset{i=1}{\sum }}{\left(y_{i}-f_{i}\right)}^{2}. \end{array}$$

Subtype classification of omics data

(12) $$\begin{array}{c} \text{MAPE}=\frac{1}{n}\overset{n}{\underset{i=1}{\sum }}\left|\frac{y_{\text{i}}-y_{i}^{\prime }}{y_{i}}\right|. \end{array}$$

Multiomics data fusion

(13) $$\begin{array}{c} \text{MAE}=\frac{1}{n}\left(\overset{n}{\underset{i=1}{\sum }}\left|y_{i}-y_{i}^{\prime }\right|\right). \end{array}$$

Subtype classification results

(14) $$\begin{array}{c} A_{H}\left(\varphi \right)=-\min\left[12{\left(\frac{\varphi }{\varphi_{3dB}}\right)}^{2},A_{m}\right]. \end{array}$$

Category division

(15) $$\begin{array}{c} A_{v}\left(\theta \right)=-\min\left[12{\left(\theta -\frac{\theta_{e\text{tilt}}}{\theta_{3dB}}\right)}^{2},{\text{SLA}}_{v}\right],\\ A\left(\varphi ,\theta \right)=-\min\left\{-\left[A_{H}\left(\varphi \right),A_{v}\left(\theta \right)\right],A_{m}\right\}. \end{array}$$

## 4. Simulation Experiment

### 4.1. Big Data Analysis of Liver Cancer Sequencing Results

The coding of the multilevel grid adopts a simple construction by assuming that the attributes of a given target value are conditionally independent of each other. It can realize the space filling of the data dimensionality reduction map, and then learn the joint probability distribution from the input to the output from the training data set. In the calculation process, it is represented by binary values 0 and 1, and input the feature data set of the unknown category to obtain the output category vector that maximizes the posterior probability. Indexing is also commonly used in Geohash encoding algorithms. There are shown in Table 1, Figures 3 and 4. The assumption that the attributes are independent of each other reduces the classification effect of the algorithm to a certain extent. According to the idea of multilevel grid, the mapping from high-dimensional space to one-dimensional space is one-to-one. The complexity is greatly simplified by encoding the one-dimensional grid of the hierarchical grid. The logic of the algorithm is relatively simple, and it also has a very stable classification efficiency. The grid division and coding rules are all calculated from the grid definition. The calculation process is to bisect the longitude values of the grid, and the data sets containing missing values are not sensitive.

### 4.2. Encoding Process of Liver Cancer Data

Big data has three invisible connotations of space, time, and semantics. As shown in Table 2 and Figure 5, convert the actual spatial position of the data to the position in the global multilevel grid, so that the two-dimensional representation of the data is converted into a binary one-dimensional representation, Collect_Time = 5.15, IMEI = 4.24, LAT = 3.23, LNG = 2.32, ECI = 2.27, EARFCN = 8.64, and PCI = 5.35. It realizes the dimensionality reduction processing of data and improves the efficiency of data organization and storage. Grid coding expresses the spatial position of data, maintains the original organization method of data, and does not abstract data objects. Collect_Time = 13, IMEI = 3, LAT = 19, LNG = 20, ECI = 20, EARFCN = 13, and PCI = 2. Instead, the expression is converted again, that is, the way of grid code identification. According to the actual area range of the object, the regional characteristics of the data are expressed as grid units, and the final grid code is composed of the codes of the grid units.

### 4.3. Naive Bayes Algorithm Training on Sequencing Data

The Naive Bayes algorithm is a classification algorithm that, in a genome screening-based approach, sequenced the human genome and many model organism genomes. As shown in Table 3 and Figure 6, for data processing that is not discretized and contains missing values, M2SMF = 3, SNF = 1, PAM50 = 4, iCluster = 4, kmeans = 4, pins = 2, and MCCA = 2. It provides new opportunities for the identification of protein targets for small molecule therapeutics. With better classification results, new chemical genomics and genomics approaches link small molecules to their protein targets. Chemical proteomic methods may also facilitate the identification of protein targets, M2SMF = 8, SNF = 5, PAM50 = 5, iCluster = 10, kmeans = 5, pins = 6, and MCCA = 5. It is used for scenarios such as efficient classification of multidimensional feature data. It will favor feature data with more attribute values and use drug affinity chromatography combined with mass spectrometry and computational analysis to classify whole protein small molecule-protein interactions. In the compound-centric chemical proteomics method, which has an impact on the construction of the decision tree and the final classification effect, the molecules are fixed on a substrate to maintain their activity and improve the accuracy of the algorithm.

### 4.4. Iterative Optimization

The EM expectation-maximum algorithm is an iterative optimization algorithm followed by incubating the cell lysate of interest with an affinity matrix. Looking for parameter maximum likelihood estimates, eluted proteins were processed without gel. As shown in Table 4 and Figure 7, the comparison of the three models shows that Naive Bayes is the best model, LAML = 0.92, KIRC = 0.96, LIHC = 0.67, M2SMF = 0.71, SNF = 0.52, MCCA = 0.67, and PINS = 0.68. Each iteration consists of alternating expected and maximal steps, which are then identified and quantified by MS. An advantage of chemical proteomics is the ability to probe the entire proteome until convergence ends. In the Okumura-Hata model, LAML = 0.03, KIRC = 0.37, LIHC = 0.5, M2SMF = 0.32, SNF = 0.49, MCCA = 0.37, and PINS = 0.8. Small molecules that encounter and interact with these proteins in their natural state and environment serve as a data addition algorithm. Another advantage of this is that proteomics can be tested in any cell type or tissue of interest, guaranteeing a steady rise in parameter value estimates over an iterative process. AdaBoost model has the worst effect, LAML = 0.38, KIRC = 0.07, LIHC = 0.55, M2SMF = 0.54, SNF = 0.27, MCCA = 0.51, and PINS = 0.36. Iterative optimization can analyze the trend of information gain rate from a large number of classification algorithm data. Therefore, the decision tree model is constructed according to the selection attributes, which is the core key to solving complex problems. The top-down recursive solution is accurate and complete. The rules for mapping attribute values to categories are a series of clear instructions for solving problems.

## 5. Conclusion

In big data analysis with the rapid improvement of computer storage capacity and the rapid development of complex algorithms, the exponential growth of massive data has also made science and technology progress with each passing day. Based on omics data such as mRNA data, microRNA data, or DNA methylation data, this study uses traditional clustering methods such as kmeans, K-nearest neighbors, hierarchical clustering, affinity propagation, and nonnegative matrix decomposition to classify samples into categories, and obtained: (1) The assumption that the attributes are independent of each other reduces the classification effect of the algorithm to a certain extent. According to the idea of multilevel grid, the mapping from high-dimensional space to one-dimensional space is one-to-one correspondence. The complexity is greatly simplified by encoding the one-dimensional grid of the hierarchical grid. The logic of the algorithm is relatively simple, and it also has a very stable classification efficiency. (2) Convert the two-dimensional representation of the data to the one-dimensional representation of binary, Collect_Time = 5.15, IMEI = 4.24, LAT = 3.23, LNG = 2.32, ECI = 2.27, EARFCN = 8.64, and PCI = 5.35. It realizes the dimensionality reduction processing of data and improves the efficiency of data organization and storage. The grid coding expresses the spatial position of the data, maintains the original organization method of the data, and does not make the abstract expression of the data object. (3) For data processing that is not discretized and contains missing values, M2SMF = 3, SNF = 1, PAM50 = 4, iCluster = 4, kmeans = 4, pins = 2, and MCCA = 2. It provides a new opportunity for the identification of protein targets of small molecule therapy and obtains a better classification effect. Chemical proteomics methods may also facilitate the identification of protein targets, M2SMF = 8, SNF = 5, PAM50 = 5, iCluster = 10, kmeans = 5, pins = 6, and MCCA = 5, for multidimensional feature data analysis. It will favor feature data with more attribute values. (4) The comparison of the three models shows that Naive Bayes is the optimal model, LAML = 0.92, KIRC = 0.96, LIHC = 0.67, M2SMF = 0.71, SNF = 0.52, MCCA = 0.67, and PINS = 0.68. Each iteration consists of alternating expected and maximal steps, which are then identified and quantified by MS. An advantage of chemical proteomics is the ability to probe the entire proteome until convergence ends.

## Figures and Tables

**Figure 1:** Conceptual model.

**Figure 2:** Screening process.

**Figure 3:** Differences in the expression of hepatocellular carcinoma-related genes.

**Figure 4:** Expression data.

**Figure 5:** Test point properties.

**Figure 6:** Classification algorithm training.

**Figure 7:** Algorithm optimization.

**Table 1:** Differences in the expression of hepatocellular carcinoma-related genes.

Gene	GeneBank	LogFC	FDR	Gene	GeneBank	LogFC	FDR
CXCL11	NM_005409.5	1	2.51	IDO1	NM_002164.6	4	2.44
KLK3	NM_001648.2	10	2.07	SLAM	NM_020125.3	2	2.01
WARS	NM_004184.4	2	2.8	OLFM	NM_006418.5	8	2.48
GBP4	NM_052941.5	8	2.77	APOC1	NM_001645.5	10	2.02
CD300LF	NM_139018.5	2	2.29	KRT81	NM_002281.4	8	2.22
ZNF683	NM_001114759.3	9	2.61	FCGR1B	NR_164759.1	5	2.06
CXCL10	NM_001565.4	8	2.35	OR2B2	NM_033057.2	7	2.8
LAM	NM_014398.4	3	2.98	CETN1	NM_004066.3	10	2.78
GBP5	NM_052942.5	1	2.9	RUNX1	NM_001754.5	5	2.65
ELANE	NM_001972.4	3	2.69	DNASE2B	NM_021233.3	4	2.29
EPSTI1	NM_001002264.4	8	2.35	IFI30	NM_006332.5	3	2.1
HAPLN3	NM_001307952.2	9	2.6	DM	NM_021951.3	1	2.02

**Table 2:** Test point properties.

	EARFCN_1	PCI_1	RSRP_1	EARFCN_2	PCI_2	RSRP_2
Collect_Time	2.32	12.13	12	5.15	13	9
IMEI	2.45	3.37	15	4.24	3	4
LAT	2.79	18.84	11	3.23	19	5
LNG	2.52	10.18	14	2.32	20	4
ECI	2.55	11.95	15	2.27	20	19
EARFCN	2.52	13.83	17	8.64	13	10
PCI	2.31	7.31	17	5.35	2	3
RSRP	2.63	6.85	14	9.77	19	17

**Table 3:** Classification algorithm training.

	CRS	EPSG	Extent	Level
M2SMF	3	8	15	2.43
SNF	1	5	14	7.86
PAM50	4	5	15	2.15
iCluster	4	10	16	4.71
kmeans	4	5	13	5.44
pins	2	6	17	2.59
MCCA	2	5	12	7.63

**Table 4:** Algorithm optimization.

	Naive Bayes	Okumura-Hata	AdaBoost
LAML	0.92	0.03	0.38
KIRC	0.96	0.37	0.07
LIHC	0.67	0.5	0.55
M2SMF	0.71	0.32	0.54
SNF	0.52	0.49	0.27
MCCA	0.67	0.37	0.51
PINS	0.68	0.8	0.36

## Data Availability

The experimental data used to support the findings of this study are available from the corresponding author upon request.
